# Macular and Optic Disc Parameters in Children with Amblyopic and Nonamblyopic Eyes under Optical Coherence Tomography Fundus Images

**DOI:** 10.1155/2022/9409749

**Published:** 2022-06-15

**Authors:** Dan Zhu, Qiang Sun, Hong Yang, Yangcheng Zou, Chunmei Liu, Yan Xu

**Affiliations:** Department of Ophthalmology, Daping Hospital, Army Medical Center, Army Medical University, No. 10, Changjiang Branch, Daping, Yuzhong District, Chongqing 400042, China

## Abstract

The aim of this study was to investigate the characteristics of macular and optic disc parameters in children with amblyopic and nonamblyopic eyes, using fundus images under optical coherence tomography (OCT). 36 patients with anisometropic amblyopia were selected in the experimental group, and another 36 healthy volunteers were selected in the control group, OCT examinations were performed in all groups, and the mean diopter, mean corrected visual acuity (CVA), mean axial length, mean optic disc retinal nerve fiber layer (RNFL) thickness, and mean macular fovea thickness were recorded in the two groups. The results found that the average diopter of the patients in the control group and the experimental group was +2.30 ± 2.54 D and +5.51 ± 1.76 D, respectively. The average CVA was 0.86 ± 0.07 and 0.22 ± 0.16, respectively; the average eye axial length was 22.41 ± 1.20 mm and 21.11 ± 0.78 mm, respectively. As *P* < 0.05, the differences were statistically significant in the three indicators between the two groups. There was no significant difference between the two groups in the average thickness of the RNFL of the optic disc and the average thickness of the central fovea of macula (*P* > 0.05). There was some correlation among CVA, diopter, eye axial length, RNFL thickness, and average thickness of macular fovea, but the correlation was not significant. It was suggested that there were certain differences in the macular and optic disc parameters between amblyopic and nonamblyopic children, but the difference is little. Thereout, a certain objective basis was provided for the early detection and treatment of amblyopia.

## 1. Introduction

Amblyopia is a common eye disease in children with impaired visual function. Infants and young children have impaired visual function due to various reasons in the perception, movement, conduction, and visual center. They cannot receive appropriate visual stimulation, thereby affecting visual development, with the main manifestations of low vision and unilateral functional impairment of both eyes [1, 2]. Amblyopia can be classified into anisometropic amblyopia, ametropic amblyopia, strabismic amblyopia, form deprivation amblyopia [3]. Its incidence is as high as 2%-4%, closely related to visual development [4]. The pathogenesis of amblyopia is very complex. Some researchers have indicated that its pathogenesis lies in the interaction of binocular abnormalities and sensory deprivation, but its histological changes are not very clear [5, 6]. There are two theories currently. The central generation theory believes that the main damaged parts of the visual pathway in patients with amblyopia are the visual cortex and the lateral geniculate body. The decline in visual input causes problems in the development of neurons in both eyes, which result in amblyopia. This theory has been widely accepted by laboratories, and it has been demonstrated that the level and activation range of the visual cortex of the amblyopic eyes are lower than those of the normal eyes [7, 8]. The peripheral theory indicates that insufficient stimulation to the retina and immaturity of the tissue structure during the sensitive period of visual development are the mechanisms of amblyopia [9]. Whether and how amblyopia alters retinal structure is still a controversial issue and a hot topic of current research.

The macula is located 0.35 cm below the temporal side of the optic disc in the fundus, is the projection point of the visual axis, and is also in the optical center of the human eye. The macula is slightly darker than the adjacent retina due to the abundance of lutein. In the center of the macula is a recessed area called the fovea, where vision is most sensitive [10, 11]. The optic disc, also known as the papilla of optic nerve, is in a reddish disc-like structure with a diameter of about 1.5 mm. It is a structure with a clear boundary from the macula to the site about 3 mm from the nasal side of the retina [12]. Previous researches have shown that there are retinal abnormalities in amblyopia patients, but a large number of subsequent studies have denied this statement. With the continuous development of medical technology, many advanced clinical instruments have been used in the auxiliary diagnosis of amblyopia in recent years, confirming that patients with amblyopia have organic changes. However, it is believed that there is no lesion in the tissue structure before [13]. Therefore, whether there is an abnormality in the retina of an amblyopia patient needs to be discussed through further experiments.

Optical coherence tomography (OCT) is a medical technique to measure the structure of living tissues. It is similar to the technique of optical microscopy for biopsied tissue in histopathology, but it is performed directly on the human body rather than obtaining the specimen surgically [14]. It has been reported that compared with the normal retinal structure, OCT imaging has a good correlation when presenting the fundus of normal patients. The resolution can reach 10 *μ*m in terms of the thickness of the retinal nerve fiber layer (RNFL), the morphological characteristics of the optic disc, and the layered structure of the retina [15]. Some scholars have found that the accuracy of retinal full thickness measured by OCT goes with a coefficient of variation of 0.05, and the correlation coefficient between the accuracy obtained by OCT measurement and that obtained by optical microscopy is 0.98. This makes OCT, as a new method of retinal imaging, be proved with the high resolution and noncontact and noninvasive characteristics [16]. Factors like refraction, axial eye, and light intensity will not affect it, so the OCT has very good reproducibility and very high reliability. In contrast to fundus photography, it can be applied to measure not only lateral but also axial images [17]. Therefore, 36 cases of anisometropic amblyopia patients (experimental group) and another 36 healthy volunteers (control group) were collected for OCT examination. OCT fundus images were taken to evaluate the foveal structure and optic disc parameters of amblyopic children and nonamblyopic children, and the possible differences between the two were analyzed. It was to provide a theoretical basis for studying the pathogenesis of amblyopia.

## 2. Materials and Methods

### 2.1. General Information

In this study, 36 amblyopia children who visited the outpatient department for the first time from May 2021 to October 2021 were included in the experimental group. 14 male patients and 22 female patients were included, aged between 6 and 18 years, and the average age was 12.56 ± 2.72 years. For amblyopia grading, 14 cases were with mild symptoms, 17 cases were with moderate symptoms, and 5 cases were severe. Another 36 healthy children who visited the clinic during the same period were selected as the control group. There were 16 males and 20 females, 13.17 ± 2.83 years old on average. As no significant difference was discovered in general clinical data between the two groups of patients, there was comparability. The two groups of children and their guardians had fully understood the situation and signed informed consent, and this study had been approved by the medical ethics committee of the hospital.

The definition of amblyopia was in line with the criteria of strabismus and amblyopia diagnostic experts as well as the Ophthalmological Society of Chinese Medical Association in 2011. It was defined that, due to various reasons, the best-corrected visual acuity of one eye or both eyes was less than the corresponding visual acuity of the age. Otherwise, if the difference in visual acuity between the two eyes was greater than or equal to 2 lines, then the eye with relatively low visual acuity was regarded with amblyopia [18]. The anisometropic amblyopia was defined as the amblyopia caused by the relatively higher diopter in an eye, with a diopter difference of 1.00 DC in binocular cylinders or that of 1.50 DC in binocular hyperopic spherical lenses [19]. The inclusion criteria were as follows. Patients underwent no treatment, including physical treatment and drug treatment. Patients had no congenital or hereditary lesions. Those with anisometropia showed a diopter of not less than 1.5 DC. They could fully cooperate with OCT and other examinations during the research period. The exclusion criteria included the following conditions. Patients had a history of eye diseases, visual pathway neurological disease, or complication with nystagmus, ptosis, leukoplakia, papillitis, glaucoma, cataract, and other diseases. They had a history of eye surgery.

### 2.2. Routine Eye Examination

All patients included were examined by the same professional ophthalmologist. The examination items included visual acuity, eye movement, eye refraction (mydriasis was performed with compound topiramate before the examination), intraocular pressure measurement, and eye axis examination. According to the CVA, amblyopia could be classified into three grades. When the corrected distance vision was 0.8-0.6, it belonged to mild amblyopia. The corrected distance vision was 0.5-0.2, which was determined as moderate amblyopia. If the corrected distance visual acuity was less than or equal to 0.1, it was severe amblyopia. The vision chart used in the examinations was in the international standard.

### 2.3. Amblyopia Treatment

The amblyopia patients were treated by wearing corrective glasses that matched the individual pathological changes and near vision training by covering the dominant eye for 2 to 6 hours every day. If conditions permitted, perceptual learning could also be added. All the tests were reviewed 6 months after amblyopia treatment. The amblyopia patients who had been treated for more than 6 months were included in the efficacy statistics, to compare the differences in the parameters of the fovea before and after treatment in the effective patients. The treatment effect of amblyopia was judged according to the standards published by the National Children's Amblyopia and Strabismus Prevention and Control Group [20], which were described below. If the CVA increased to 0.8 or more, it was considered to be basically cured. If the visual acuity improved by 2 lines or more with the international standard vision chart, it was considered to be improved. If the visual acuity dropped, there was no obvious change, or the improvement did not reach 2 lines, it was ineffective; it was also judged with the international standard vision chart.

### 2.4. OCT Examination

The OCT examination was performed. When the pupil dilated to a diameter greater than 6 mm after mydriasis, the patients were asked to sit in front of the instrument, and the examination was started using the internal fixation method. The information on the macular area was obtained by the scanning method of the macular volume of 512 × 128. With the fovea as the center, the diameter of the linear scanning was 1 mm, 3 mm, and 6 mm, respectively. There were 6 radial scanning lines in total, each with an included angle of 30°. The scanning results of each eye at the fovea were automatically displayed by the instrument analysis software, including the retinal thickness and retinal thickness/volume analysis. The scanning parameters of each eye were the same. The information around the optic disc was acquired using the optic disc cube 200 × 200 scanning method, and the average thickness of the RNFL around the optic disc was automatically displayed by the built-in analysis software of the instrument. The average macular thickness and macular volume of the patients in the experimental group were observed and recorded before and after treatment, and the disc edge area, the average cup/disc diameter ratio (C/D), the average vertical C/D, and the optical cup volume were also recorded.

### 2.5. Observation Indicators

The macular parameters (average foveal thickness and retinal volume in central macular area) and optic disc parameters (average fiber layer thickness of peripheral nerve around the optic disc, disc edge area, average C/D, average vertical C/D, and optic cup volume) were observed and recorded in both groups. The clinical treatment effect of the patients in the experimental group was also observed and recorded, and the correlation among the indicators was analyzed.

### 2.6. Statistical Analysis

SPSS 19.0 was used for statistical processing of the obtained data, and the measurement data were expressed as the mean ± standard deviation ($\bar{x}\pm s$). Differences in foveal thickness, average RNFL thickness around the optic disc, and macular volume were compared between children with amblyopia and normal children through the paired *t*-test. The Pearson correlation analysis method was adopted to analyze the correlation among the eye axial length, the average foveal thickness, macular volume, RNFL thickness around the optic disc, optic disc area, and other optic disc parameters in the two groups. When *P* < 0.05, the difference was considered statistically significant.

## 3. Results

### 3.1. General Conditions of the Two Groups of Patients

After measurement, the average CVA of the patients in the control group and the experimental group were 0.86 ± 0.07 and 0.22 ± 0.16, respectively. The average diopter was +2.30 ± 2.54 D in the control group and +5.51 ± 1.76 D in the experimental group. The average eye axial length was 22.41 ± 1.20 mm and 21.11 ± 0.78 mm, respectively, and the differences of the three indicators were statistically significant, *P* < 0.05. It is shown in Figure 1 for details.

### 3.2. Comparison of Macular Parameters between the Two Groups

The average thickness of the central fovea of macula in the experimental group was 285.79 ± 8.24 *μ*m, and that in the control group was 283 ± 7.12 *μ*m. There was no significant difference in the thickness between the two groups, *P* > 0.05. The average retinal volume in the central macular area was 11.36 ± 0.17 mm^3^ for patients in the experimental group, while that in the control group was 11.13 ± 0.23 mm^3^. No significant difference was found in the retinal volume between the two groups, *P* > 0.05; details are presented in Figure 2.

The average foveal thickness and macular retinal volume were compared in patients with amblyopia in different degrees in the experimental group. There were only 5 patients with severe amblyopia in the group, and the macular parameters were not compared with those of mild and moderate amblyopia patients. There was no significant difference in the average foveal thickness and macular retinal volume between patients with mild and moderate amblyopia, *P* > 0.05.  Figure 3 displays the details.

Among 36 patients in the experimental group after treatment, 23 cases with amblyopia were reexamined on time after comprehensive treatment for 6 mo. Among them, 4 patients were basically cured (17.4%), 13 patients were improved (56.5%), and the effect in 6 patients was thought to be ineffective (26.1%). The total effective rate was 73.9%. There were 17 cases with effective treatment, and no significant difference was observed in the parameters of the fovea of their amblyopic eyes before and after treatment by OCT, *P* > 0.05. The details are presented in Figures 4 and 5.

### 3.3. Comparison of Optic Disc Parameters between the Two Groups of Patients

The average RNFL thicknesses of the experimental group and the control group were 98.77 ± 2.93 *μ*m and 99.76 ± 3.84 *μ*m, respectively. The disc edge area, average C/D, average vertical C/D, and optic cup volume were compared between the two groups, and no significant difference was discovered with *P* > 0.05. It is shown in Figures 6 and 7 for details.

### 3.4. Correlation Analysis

From the correlation analysis among various indicators of amblyopia patients, it was found that the eye axis and the thickness of the fovea as well as the thickness of the RNFL around the optic disc were negatively correlated. The *P* values were 0.35 and 0.21, respectively; thus, the correlation was not of significance. The diopter was positively correlated with the thickness of the fovea and the thickness of the RNFL, and the *P* values were 0.23 and 0.11, respectively; the correlation was not obvious. The best CVA was negatively correlated with the two thicknesses, with the *P* values of 0.78 and 0.58, respectively. Therefore, it could be observed that the correlation was not significant, as the details are in Figures 8 and 9.

## 4. Discussion

OCT is realized by the computerized tomography of near-infrared light scanning, which can identify the microscopic structure of the retina. OCT has the advantages of high resolution, noncontact, and noninvasion and is not affected by factors such as refraction, axial eye, and light intensity, with high reproducibility and high reliability [21, 22]. Using this technique, the microstructure of the retina in vivo can be obtained. Since 2016, OCT has been applied more and more widely, as it automatically locates and precisely measures the distance between the inner limiting membrane and the retinal pigment epithelium at a speed of 20,000 scans per second [23]. Some scholars have utilized animal experiments to prove that the retinal thickness measured by OCT is basically the same as the value measured by the histological method. Furthermore, with the increase in an animal's age, the trends of these two changes are also consistent [24].

Kausar et al. [25] applied OCT to examine 26 patients with persistent amblyopia and 25 patients with cured amblyopia. By comparing the RNFL thickness of persistent amblyopia, cured amblyopia, and normal contralateral eye, it was found that there was no statistically significant difference among the RNFL thicknesses of persistent amblyopia, cured amblyopia, and the normal contralateral eye. Logistic regression analysis of adjusted diopter showed no significant difference in RNFL thickness between persistent amblyopia and cured amblyopia. Therefore, the thickness of the RNFL did not differ significantly between amblyopic and nonamblyopic patients. On the contrary, Zhang et al. [26] studied the average thickness of binocular optic disc RNFL in monocular amblyopic patients by OCT detection technology and found that there were certain differences in the structure of RNFL around the optic disc monocular amblyopic patients and nonamblyopic patients. The OCT imaging technique was used to observe the macular thickness of patients with anisometropic amblyopia here and to compare the difference between it and nonamblyopia patients. It was suggested that there was no statistically significant difference in the average thickness of the fovea between the two groups. The retinal volume in the central area of the macula in patients with amblyopia was larger than that in nonamblyopic patients, but the difference was also not statistically significant. These were similar to the research results of some scholars in the world [27].

There was no statistically significant difference in the average foveal thickness and macular volume between patients with mild and moderate amblyopia. This is similar to the findings of Nagai et al. [28]. Six months after comprehensive treatment for amblyopia, the total effective rate of 23 patients was 73.9%. No significant difference was observed in the macular fovea indicators before and after treatment. The results suggested that retinal development in patients with amblyopia might be slower than vision improvement, which was similar to that of Batum et al. [29]. With the increase in treatment time, the development of the retina in the amblyopic macular region and the changes in OCT parameters in the fovea needed to be further studied and observed.

Some scholars used OCT technology to examine the RNFL around the optic disc, with 38 patients with strabismus and anisometropic monocular amblyopia as the research objects. They find that the average RNFL thickness of amblyopia is significantly thicker than that of normal eyes. After grouping according to the types of amblyopia, there is still a significant difference between refractive error and anisometropic amblyopia, as the difference in the RNFL structure around the optic disc is taken into consideration between amblyopic patients and nonamblyopic patients [30]. The average RNFL thickness around the optic disc in patients with anisometropic amblyopia was observed by OCT imaging here and was compared with that in nonamblyopic patients. No statistically significant difference was shown in the average thickness of the RNFL around the optic disc between the two groups, and the differences in the parameters of the optic disc were also not statistically significant.

Given the possible relationship between the three indicators of best CVA, eye axial length, and diopter and the thickness of the RNFL around the optic disc as well as the thickness of the fovea, a correlation analysis was conducted. It was suggested that the eye axis had a negative correlation with the thicknesses of the fovea and the RNFL; for the *P* value was 0.35 and 0.21, the correlation was not remarkable. The relationship between the diopter and the two thicknesses was positively correlated; the *P* value was 0.23 and 0.11, respectively; so, the correlation was not significant. The relationship between the best CVA and the thicknesses was negatively correlated; as the *P* values were 0.78 and 0.58, respectively, the correlation was not obvious. Therefore, the role of nonvisual factors might affect the thickness of the RNFL, which was very inconsistent with the results of many foreign researches [31]. This may be influenced by racial differences or some subjective and objective factors, such as the degree of cooperation between patients, differences between individuals, and the size of the experiment sample. All of these factors needed to be verified via further exploration.

## 5. Conclusion

OCT fundus images were used for evaluating the macular parameter characteristics and optic disc parameter characteristics of amblyopic and nonamblyopic children in this work. There were significant differences in the average diopter, average corrected visual acuity, and average eye axis between the control group and the experimental group. No significant difference was shown in the average fiber layer thickness of the peripheral nerve around the optic disc as well as the average foveal thickness. There was a certain correlation among the corrected visual acuity, diopter, axial and retinal nerve fiber layer thickness, and the average foveal thickness, but it was not significant. It was also necessary to consider the developmental characteristics of the retina in amblyopic eyes and the pathogenesis of amblyopia in the future. An in-depth comprehensive analysis could be conducted combined with multiple clinical factors and larger samples. This work provided some theoretical references for the mechanism research of amblyopia.

## Figures and Tables

**Figure 1:** General situation of patients in the two groups. # meant *P* < 0.05, as the differences were statistically significant.

**Figure 2:** Comparison of the average thickness and total retinal volume of the macular fovea between the two groups.

**Figure 3:** Comparison of macular parameters in patients with mild and moderate amblyopia in the experimental group.

**Figure 4:** Evaluation of the treatment effect on patients in the experimental group.

**Figure 5:** Comparison of macular parameters before and after treatment in the experimental group.

**Figure 6:** Comparison of the average thickness of the RNFL around the optic disc of patients between the two groups.

**Figure 7:** Comparison of optic disc parameters between the two groups.

**Figure 8:** Correlation analysis between indicators and foveal thickness in patients with amblyopia.

**Figure 9:** Correlation analysis between indicators and the thickness of RNFL around the optic disc in patients with amblyopia.

## Data Availability

The data used to support the findings of this study are available from the corresponding author upon request.
